This article has been retracted.

# Severe Dengue With Multisystem Inflammatory Syndrome in Children Due to COVID-19: A Co-infection Case Series

**DOI:** 10.7759/cureus.19516

**Published:** 2021-11-12

**Authors:** Anima Ferdous, M Monir Hossain, Manifa Afrin

**Affiliations:** 1 Pediatric Intensive Care Unit, Universal Medical College Hospital, Dhaka, BGD; 2 Pediatric Medicine, Universal Medical College Hospital, Dhaka, BGD

**Keywords:** sars-cov-2 (severe acute respiratory syndrome coronavirus -2), covid 19, mis-c in children, severe dengue, dengue with mis-c co-infection

## Abstract

Severe dengue with the multisystem inflammatory syndrome in children (MIS-C) can be difficult to diagnose as both diseases have similar symptoms and laboratory findings. Bangladesh is currently facing a double burden of severe dengue and SARS-CoV-2 infection. Co-infection with these viruses can result in severe morbidity. Worldwide this co-infection is rare. However, we present five cases of severe dengue with possible MIS-C due to SARS-CoV-2 infection in children. All the children presented with shock with variable degrees of plasma leakage. Mucocutaneous and gastrointestinal involvement were common. All tested positive for dengue nonstructural protein 1 antigen on the second to the third day of fever and tested positive for anti-SARS-CoV-2 IgG by enzyme-linked immunosorbent assay. Echocardiographic evaluation in all patients showed coronary arterial abnormalities. Cardiac enzymes were abnormal, and there were raised inflammatory markers and abnormal coagulation profiles. One patient had neurological involvement and needed mechanical ventilatory support. All cases were successfully managed according to dengue shock syndrome guidelines and required intravenous immunoglobulin with prednisolone, aspirin, and in some cases, enoxaparin for the management of coronary arterial involvements, which is not a documented feature for severe dengue infection, but typically found in MIS-C due to SARS-CoV-2 infection or Kawasaki disease. This case series aims to describe the possibility of co-infection of severe dengue with MIS-C due to SARS-CoV-2 infection in a dengue-endemic region during the coronavirus disease 2019 (COVID-19) pandemic, and alternatively, dengue virus as an unusual etiology for Kawasaki disease was also entertained. Severe dengue in endemic regions can coexist with COVID-19 during an outbreak, making it hard to diagnose. It can be fatal without early, appropriate management.

## Introduction

In December 2019, the severe acute respiratory syndrome coronavirus 2 (SARS-CoV-2) was first identified in Wuhan, China. Its spread has resulted in a pandemic since then [1]. The SARS-CoV-2 pandemic has resulted in a novel set of clinical manifestations called pediatric inflammatory multisystem syndrome-temporally associated with SARS-CoV-2 (PIMS-TS) in Europe or multisystem inflammatory syndrome in children (MIS-C) by the World Health Organization (WHO) and in the USA [1-3]. Several studies described clusters of children and adolescents with SARS-CoV-2 infection presenting with an acute illness accompanied by a hyperinflammatory syndrome, leading to multiorgan failure and shock. The features are like those of Kawasaki disease or toxic shock syndrome [2-5].

Amidst the SARS-CoV-2 pandemic, Southeast Asia is also experiencing a dengue virus outbreak. Dengue fever is the most rapidly spreading mosquito-borne viral disease worldwide with an unpredictable clinical course [6-8]. Most cases are usually mild and do not require hospitalization; however, some patients develop severe complications, including shock, bleeding manifestations, encephalopathy, hepatic failure, renal failure, cardiac arrhythmia, and myocarditis [7]. Co-infection with both viruses poses a major health problem. This case series aims to demonstrate cases with possibilities of simultaneous severe dengue and MIS-C due to COVID-19; alternatively, dengue virus as an unusual etiology for Kawasaki disease was also entertained. Missing a case due to the overlapping symptoms and signs, pathological similarities, and immunological cross-reactivity can lead to a fatal outcome. To the best of our knowledge, this is the first case series from Bangladesh demonstrating severe dengue and MIS-C in pediatric patients, with MIS-C due to SARS-CoV-2 confirmed by enzyme-linked immunosorbent assay (ELISA).

The information in this clinical case series was obtained through clinical record review and interviews. All patients tested positive for dengue nonstructural protein 1 antigen (NS1 Ag) (sensitivity 55%-82% and specificity 97%-100%) [6,7] and partially fulfilled WHO’s criteria for MIS-C [1]. Though during the inclusion, the patients had dengue NS1 Ag positive, other microbiological causes were excluded, as guided by WHO for diagnosis of MIS-C in children due to COVID-19. Included cases either had an obvious history of flu-like symptoms or features of upper respiratory tract infection within three weeks prior to the presenting complaints or close, household contact with positive reverse transcription-polymerase chain reaction (rt-PCR) for COVID-19 cases within one month and positive serology for antibody (IgG) for SARS-CoV-2 by ELISA, which gave the important clue regarding the timing of performing rt-PCR for SARS-CoV-2 and the negative results. Inadequate contact tracing, awareness among the people of Bangladesh can be an important issue here. Some studies stated that only 70% of pediatric MIS-C cases due to COVID-19 were PCR positive [9]. Thus, diagnoses for MIS-C were made using positive serology. 

Due to immunological cross-reactivity, patients who were dengue IgM positive along with anti-SARS-CoV-2 antibody (IgG) positive were not included. Kawasaki disease, macrophage activation syndrome, and severe septicemia were the differential diagnoses. However, the patients did not fulfill the criteria for classical Kawasaki disease or macrophage activation syndrome, and blood, urine, and throat swab cultures were also negative. Dengue virus as an unusual etiology for Kawasaki disease was considered.

## Case presentation

Case 1

A four-year-old, previously healthy boy weighing 24 Kg, from Dhaka, was admitted with a four-day history of a high continued fever. He also complained of suffering abdominal pain, loose motions, and emesis for two days. He had no history of flu-like symptoms, cough, or respiratory distress in the past month. There was a history of close contact with a COVID-19 patient (within one month of the illness). He had no history of dengue. On examination, he was found febrile (temperature 102°F), tachypneic, and tachycardic with unrecordable blood pressure. Auscultation of lungs revealed bilateral crepitations with good air entry. The abdomen was distended, flanks were full with mild, diffuse abdominal tenderness. Initial investigations showed dengue NS1 Ag positive and rt-PCR for SARS-CoV-2 negative, thrombocytopenia, positive C-reactive protein, altered coagulation profiles (Table 1).

**Table 1:** Investigation profile of cases NT-pro = N-terminal-pro hormone

Investigations	Reference range	Case 1	Case 2	Case 3	Case 4	Case 5
Dengue nonstructural protein 1 antigen (NS1 Ag)		+	+	+	+	+
Anti-SARS-CoV-2 IgG (ELISA)		+	+	+	+	+
Complete blood count						
Hemoglobin (g/dl)	Male, 12-17; female, 11.5-15.5	10	14	9.6	9.1	15.4
Hematocrit (%)	Male, 40-52; female, 36-48	31	42	29	28.2	44.4
Total WBC (10^9^/L)	4-11	4.9	6.98	5	4.6	10.6
Neutrophils (%)	40-75	56	77	17	45	34
Platelet count (10^9^/L)	150- 450	55	25	32	32	42
C-reactive protein (mg/dL)	0.01-0.30	3.16	5.00	7.66	3.02	1.21
Serum procalcitonin (ng/mL)	<2.0	0.87	0.1	5.20	0.47	1.56
Serum albumin (g/dl)	3.4-5.0	4.15	3.17	2.75	2.17	1.8
Serum calcium (mg/dl)	8.20- 10.20	9.3	7.8	7.9	6.00	6.60
Alanine transferase (ALT) (U/L)	<40	30	97	35	30	578
Aspartate aminotransferase (AST) (U/L)	<37	70	168	92	78	180
Prothrombin time (PT) (sec)	Control- 12	14	14	12	16	17
Activated partial thromboplastin time (APTT) (sec)	Control- 28	72	36	34	55	53
Blood urea (mg/dl)	10-40	30	12	10	10	41
Serum creatinine (mg/dl)	0.2-0.7	0.58	0.78	0.42	0.67	0.84
Serum ferritin (ng/ml)	7-140	Before treatment: >2000 After treatment: 432	Before treatment: >2000	Before treatment: 595	Before treatment: 2000 After treatment: 950	Before treatment: >2000 After Treatment: 980
D-dimer (mg/L)	<0.5	Before treatment: >5	Before treatment: >5 After treatment: 1.35	Before treatment: >5 After treatment: 2.7	Before Treatment: 5 After treatment: 0.37	Before Treatment: >5 After treatment: 2.3
NT-pro-B-type natriuretic peptide (pg/ml)	<125	Before treatment: 8953 After treatment: 2058	Before treatment: 1550 After treatment: 383	Before treatment: 3730 After treatment: 2031	Before treatment: 390 After treatment: 140	Before treatment: 9432 After Treatment: 5022
Serum troponin I (ng/ml)	0.00-0.056	Before treatment: 1.844 After treatment: 0.430	0.00	Before treatment: 0.579 After treatment: 0.019	Before treatment: 0.017 After treatment: 0.00	Before treatment: 0.485 After treatment: 0.30

The chest X-ray (CXR) initially revealed bilateral pulmonary infiltrations. He was treated for dengue shock syndrome with plasma leakage with intravenous (IV) ceftriaxone, inotropes, and colloids. On the 5th and 6th day of fever, he developed petechial rashes on both extremities, cheilosis, and an erythematous rash over the trunk (Figure 1). 

**Figure 1:** An image of the trunk of Case 1 The blue arrow shows erythematous maculopapular rash on the trunk

The patient also developed a cough and respiratory distress, oxygen saturation (SpO_2_) by pulse oximeter was found to be 96% with 5L/min oxygen through a face mask. Repeat CXR revealed bilateral inflammatory lesions with pleural effusion. The ECG was normal. However, echocardiography revealed dilated coronary arteries, left main coronary artery (LMCA, +3.0 standard deviation, SD), left coronary artery (LCA, +2.5 SD) with the loss of distal tapering and mild left ventricular (LV) dysfunction (ejection fraction [EF] 52%) (Figure 2).

**Figure 2:** Echocardiogram of Case 1 The image shows dilated coronaries with loss of distal tapering and mild left ventricular dysfunction (ejection fraction, 52%)

Initial serum ferritin, N-terminal-pro hormone B-type natriuretic peptide (NT-pro-BNP), D-dimer, serum troponin I were markedly raised (as shown in Table 1). The anti-SARS-CoV-2 antibody (IgG) test came back positive on the seventh day of fever. A pediatric cardiologist was consulted, and we administered one dose of intravenous immunoglobulin (IVIG) 2 g/Kg, along with enoxaparin 2 mg/Kg for five days. Thereafter, oral prednisolone and aspirin were added. Meanwhile, the patient became afebrile, and the rash faded. His general condition improved with a gradual return of appetite. Three days after the IVIG, repeat tests showed decreasing serum ferritin, NT-pro-BNP, and serum troponin I. The patient was transferred to the ward after 12 days in the pediatric intensive care unit (PICU) thereafter discharged after five days with the necessary advice and follow-up appointment.

Case 2

A previously healthy 12-year-old girl from Dhaka, weighing 55 Kg, was admitted with a four-day history of high intermittent fever, headache, arthralgia, and generalized body aches. She had an erythematous rash on her trunk, cough, and respiratory distress. She was initially admitted to another hospital, but her condition deteriorated, and she developed shock and was referred to our PICU. She had complained of flu-like symptoms within two weeks of the presenting illness. She had a history of one episode of dengue fever three years earlier but no contact history with a COVID-19 patient.

On admission, the patient was conscious, febrile (temperature 104°F), tachypneic, tachycardic with unrecordable blood pressure, and prolonged capillary refill time. SpO_2_ by pulse oximeter was 93% in room air and 96% with 2L/min oxygen via nasal cannula. Auscultation of lungs revealed bilateral diminished air entry with coarse crepitations, pleural rub. The abdomen was distended, full flanks with diffuse mild tenderness. She tested dengue NS1 Ag positive on the second day of fever. Management for dengue shock syndrome with plasma leakage was initiated with inotropes, IV furosemide, and albumin along with IV ceftriaxone and amikacin. She was given oxygen 3L/min via a face mask. The initial investigations showed thrombocytopenia, mild hypoalbuminemia, hypocalcemia, positive C-reactive protein, altered liver function tests with coagulopathy (as given in Table 1). Her chest X-ray showed bilateral pleural effusions with pneumonitis (Figure 3).

**Figure 3:** Chest X-ray of Case 2 Blue arrows show bilateral pleural effusion and yellow arrows show bilateral pneumonitis

A bedside echocardiogram revealed a prominent LMCA (+2.54 SD), minimal pericardial effusion, mild pleural effusion, and good biventricular function (EF 77%). Her NT-pro-BNP, serum ferritin, D-dimer were significantly high but serum troponin I was normal. At this time, the patient had mucocutaneous involvement with respiratory symptoms. Her anti-SARS-CoV-2 IgG came back positive. After reviewing the laboratory reports and echocardiographic features, we consulted the pediatric cardiologist. She was treated with one dose of IVIG 2g/Kg and started on oral prednisolone and aspirin. The patient was transferred to the main ward when she began to show clinical and laboratory improvements. She was soon discharged with the necessary advice and follow-up arrangements.

Case 3

A three-year-old girl from Dhaka, previously healthy and thriving, weighing 16 Kg, was admitted to PICU with the complaint of five days of high continued fever with diffuse, central abdominal pain, emesis, and diarrhea for the last two days. She had experienced two episodes of melena and hematemesis. She had a history of contact with a COVID-19 positive patient in the last month but had no symptoms before the present illness. There was no previous history of dengue. She had been treated in another hospital for shock, and her dengue NS1 Ag was positive on the second day of fever. On admission, the patient was febrile, with narrow pulse pressure. Her blood pressure (BP) was 60/45 mmHg with tachycardia, she had tachypnea with a SpO_2_ of 90% by pulse oximeter in room air, a low volume pulse, and cold extremities. Auscultation of lungs revealed diminished breath sound with crepitations bilaterally. The abdomen was distended and tender. She was diagnosed with dengue shock syndrome with plasma leakage. She was treated with inotropes, IV furosemide, colloids, and levofloxacin. She was given 5L/min oxygen via a face mask. Her initial investigations revealed thrombocytopenia, hypoalbuminemia, hypocalcemia, positive C-reactive protein, mildly raised serum procalcitonin, altered liver function, and coagulopathy (as shown in Table 1). Her CXR revealed bilateral pleural effusions with pneumonitis. Echocardiography showed prominent dilated coronaries, LMCA (+2.5 SD), LAD (+2.0 SD) with loss of distal tapering and perivascular brightness, bilateral pleural effusions, a mildly dilated left ventricle with mild LV dysfunction (EF 57%) (Figure 4).

**Figure 4:** Echocardiography of Case 3 Echocardiography revealed prominent coronaries, mildly dilated left ventricle, mild left ventricular dysfunction (ejection fraction, 57%)

Cardiac enzymes showed raised serum troponin I, NT-pro-BNP with raised serum ferritin and marked increased D-dimer level. The rt-PCR for SARS-CoV-2 Ag came back negative; however, the anti-SARS-CoV-2 antibody (IgG) was sent and came positive. By the sixth day of fever, the patient had conjunctival congestion and an erythematous rash on her trunk, which gradually faded (Figure 5).

**Figure 5:** An image of eyes of Case 3 Yellow arrows show bilateral conjunctival congestion

After consultation with cardiologists, one dose of IVIG 2g/Kg was given; thereafter, oral prednisolone and aspirin were added. Three days after the IVIG, repeat tests showed decreased serum troponin I and NT-pro-BNP. As her general condition had improved, the patient was transferred to the pediatric ward after seven days of PICU support. Thereafter she was discharged with advice and a follow-up appointment.

Case 4

A previously healthy nine-year-old boy, weighing 37 Kg, and hailing from Dhaka, was admitted to PICU with a high, continued fever that had lasted four days. He suffered with a headache and generalized body aches for two days and diffuse abdominal cramps with diarrhea and emesis for one day. He had a history of an upper respiratory tract infection three weeks earlier but had not done an rt-PCR for SARS-CoV-2 Ag during that time. He had no obvious contact history with a COVID-19 patient and no history of dengue infection. He tested positive for dengue NS1 Ag on the third day of fever and was admitted to another hospital. After deteriorating, the patient was referred to our PICU. On admission, he had unrecordable BP, tachycardia, tachypnea, cold extremities, breath sound was absent on right side, diminished on the left chest wall with coarse crepitations, SpO_2_ 89% in room air by a pulse oximeter. The abdomen was distended, full flanks with diffuse abdominal tenderness. He was resuscitated, and management for dengue shock syndrome with plasma leakage was started. He was given 5L/min oxygen via a face mask, IV inotropes, albumin, colloids, furosemide, imipenem, and amikacin. His blood test results included anemia, thrombocytopenia, hypoalbuminemia, marked hypocalcemia, positive C-reactive protein, raised blood urea level, mild alteration of liver functions with coagulopathy (as given in Table 1). A stool occult blood test was positive. His CXR revealed pleural effusions and pneumonitis. His ECG showed sinus tachycardia. The echocardiogram performed on the second day of admission revealed minimal pericardial effusion, bilateral pleural effusions, mild LV dysfunction (EF 59%). In addition, he had high serum ferritin, D-dimer along with a slightly raised NT-pro-BNP, normal serum troponin I. Clinically, he developed an erythematous rash on his trunk with conjunctival congestion on the seventh day of fever, which warranted further anti-SARS-CoV-2 antibody testing. This came back positive on the eighth day of fever. After consultation with pediatric cardiologists, the patient was started on IV methylprednisolone at a dose of 30 mg/Kg for three days. On the ninth day of illness, the patient developed respiratory distress and became confused and aggressive. His blood pressure was still fluctuating. His SpO_2_ was about 88% with 7L/min oxygen (2L/min via nasal cannula, 5L/min through face mask). He was placed on mechanical ventilation. Repeat CXR showed persistent pulmonary infiltrations with pleural effusion (Figure 6).

**Figure 6:** Chest X-ray of Case 4 during mechanical ventilation Yellow arrows show bilateral patchy opacities with consolidation (red arrow) and pleural effusion (blue arrow)

A brain MRI revealed no obvious neurological abnormalities. Repeat echocardiography revealed dilated coronaries, LMCA (+2.6 SD), LAD (+2.5 SD), with loss of distal tapering, bilateral pleural effusion, mild LV dysfunction (EF 51%) (Figure 7).

**Figure 7:** Echocardiogram of Case 4 The echocardiogram revealed dilated coronaries with loss of distal tapering, mild left ventricular dysfunction (ejection fraction, 51%)

After consulting with a pediatric neurologist and cardiologist, one dose of 2 g/Kg IVIG was given. Methylprednisolone and aspirin were added, and we closely monitored his platelet count. From the second day on ventilatory support, he began to improve and was gradually weaned from the ventilator. After 10 days of illness, his neurological complaints started resolving, repeat blood tests results were improved with gradual remission of pleural effusion. The patient was transferred to the pediatric ward after 12 days of PICU admission. He was discharged on request after five days with the necessary advice and follow-ups.

Case 5

A nine-year-old, previously healthy, developmentally well male child, weighing 31 Kg, and hailing from Dhaka, was admitted to the PICU. He complained of high, irregular fever over the previous four days and generalized body aches, headache, abdominal cramps with emesis for the previous two days. He had a history of dengue infection two years ago and positive contact history with a COVID-19 patient one month before the illness. He tested positive for dengue NS1 Ag on the second day of fever and was admitted to another hospital. Due to respiratory distress and fluctuating blood pressure, he was referred to our PICU. On admission, the patient had low mean pressure, tachypnea, tachycardia with a cold periphery. His breath sound was diminished bilaterally and course crepitations were heard on auscultation. He was febrile with erythematous, petechial rashes on both lower limbs, and gum bleeding. His rt-PCR for SARS-CoV-2 was negative, and blood and urine cultures yielded no growth. Initial investigations revealed, thrombocytopenia, marked hypoalbuminemia, hypocalcemia, altered liver functions, coagulopathy, positive C-reactive protein, negative procalcitonin, and slightly increased blood urea. His serum ferritin, D-dimer, serum troponin I, and NT-pro-BNP were very high (as given in Table 1). The CXR revealed bilateral pleural effusions with pneumonitis (Figure 8).

**Figure 8:** Chest X-ray of Case 5 The blue arrow shows pleural effusion and the yellow arrows show bilateral patchy opacities

The ECG showed sinus tachycardia. Management of dengue shock syndrome with plasma leakage was started with IV inotropes, albumin, calcium gluconate, antibiotics (imipenem, levofloxacin), and furosemide. An echocardiogram was done and showed a mild pericardial effusion, prominent dilated coronaries, LMCA (+3.0 SD), LAD (+2.5 SD), bilateral pleural effusion, fair LV function. The test for SARS-CoV-2 antibody (IgG) came back positive. After evaluating his condition and consultation with pediatric cardiologists, a single 2g/Kg dose of IVIG was administered, followed by methylprednisolone, aspirin, and clopidogrel. His general condition gradually improved with improving laboratory reports. Serial CXRs showed gradually decreasing pleural effusions. He was transferred to the pediatric ward 10 days after PICU admission and was discharged with the necessary advice and follow-up plans.

## Discussion

Bangladesh experienced its deadliest outbreak of dengue in 2019, with 101,354 reported cases and 179 deaths [8]. Meanwhile, the worldwide burden of MIS-C due to COVID-19 in the pediatric age group is increasing according to several cohort studies [9-14].

This series describes five cases of severe dengue with a possible MIS-C due to SARS-CoV-2 co-infection admitted to our PICU. As with earlier reports, all patients were previously healthy [14]. All were positive for dengue NS1 Ag and negative for rt-PCR for SARS-CoV-2. But, as two cases had history of possible COVID-19 infections within three weeks of presenting complaints; others had close contact with COVID-19 positive patients in past one month, this timing provides possible explanation for negative rt-PCR for COVID-19. The presenting features partially fit for WHO criteria for MIS-C in children, ELISA was performed to check for IgG antibodies for SARS-CoV-2. The results were positive. Cases 2 and 5 had a positive past history of dengue fever that occurred three and two years ago, respectively, and had been admitted for treatment. Two cases were less than five years old, while the others were eight to 12 years old. There were two female cases. All lived in Dhaka, a dengue-endemic zone [8].

All the cases had experienced a high continued or intermittent fever for more than four days, which fits the WHO criteria for MIS-C due to COVID-19, but doesn't fulfill the criteria for Kawasaki disease [1,3]. Variable headache, photophobia, arthralgia, and extremity edema were observed. These symptoms are commonly observed in patients with dengue fever, though they are sometimes features of SARS-CoV-2 infection [15,16]. Patients had bleeding manifestations, probably due to severe dengue [6]. All five patients had dyspnea with pleural effusion and pneumonitis. Both dengue and MIS-C due to COVID-19 can give these features, but the CXR findings of pneumonic infiltrations were consistent with COVID-19 infections. In dengue, pleural effusions are commonly observed, not very commonly seen patchy consolidations. Abdominal pain and vomiting are common with dengue, but diarrhea is more commonly observed in covid-19 patients [16]. Conjunctival congestion occurred in cases 2 and 3, while all of them had mucocutaneous involvement, including rashes, itchy scaling, and cheilosis. It was difficult to differentiate dengue from the MIS-C rashes. Similar types of rashes are observed in both viral infections due to the pathophysiological similarities [15,16]. None had palpable lymph nodes, commonly seen in Kawasaki disease. All patients presented with shock, either on admission or during the illness, requiring fluid management according to dengue protocols [6], in addition to colloid and inotrope support. Pleural effusion was found in all patients, requiring furosemide. Profound shock and capillary leakage are common in severe dengue and MIS-C due to SARS- CoV-2 [15,16].

All five patients had the necessary laboratory workups during admission and after suspicion of MIS-C. Raised hematocrit, thrombocytopenia, and leucopenia were observed; these abnormalities settled with timely management. Dengue and SARS-CoV-2 share some pathological features such as plasma leakage, thrombocytopenia, and coagulopathies. Severe thrombocytopenia is not commonly observed in COVID-19 associated MIS-C. However, it is common during the critical phase of dengue shock syndrome [6,10,15]. All our cases showed severe thrombocytopenia, positive C-reactive protein, raised serum ferritin, altered liver function tests, and coagulopathy. Coagulopathy is one of the main pathologies associated with dengue infection but is also seen in SARS-CoV-2 infection [6,7,10,15,16]. D-dimer levels were significantly raised in all cases. In severe dengue and MIS-C, D-dimer levels seem to be increased. Evidence suggests a hypercoagulable state in COVID-19 patients, leading to pulmonary embolism, venous thromboembolism, myocardial infarction, stroke, and microvascular thrombosis [15,16]. Serum troponin I was increased in three patients, while NT-pro-BNP was significantly elevated in all patients (Table 1). On echocardiogram, all five patients had coronary arterial abnormalities, and three patients had mild LV dysfunction. In severe dengue, cardiac involvements are not uncommon including raised cardiac enzymes, sinus bradycardia, ST and T changes in ECG, global hypokinesia and reduced ventricular functions evident in echocardiogram. Cardiac involvement in dengue lead to poor prognosis [15-17]. In this case series, all patients had their echocardiographic evaluations which demonstrated coronary arterial abnormalities commonly seen in MIS-C due to COVID-19 or Kawasaki disease, but no case report to date demonstrated coronary arterial abnormalities due to dengue [5,6]. There are two possible explanations for the unusual findings in these patients: (1) concomitant severe dengue and MIS-C due to COVID-19, or (2) severe dengue as an etiology for atypical Kawasaki disease including coronary arteritis. But, as per our knowledge, no case is reported with evident coronary arterial involvement in dengue. As MIS-C due to SARS-CoV-2 is still an unknown domain and still in the phase of evolving evidence, very limited cases are coming forth regarding this co-infection, hence the possibility of co-infection of the mentioned viruses cannot be ruled out. Several studies have shown an association of raised troponin I and NT-pro-BNP with ventricular dysfunction and coronary artery abnormalities in pediatric MIS-C [9-12]. These may be an atypical Kawasaki disease, with very unusual initial presentation in the form of thrombocytopenia and plasma leakage, shock. This hypothesis is not supported by positive NS1 Ag for the dengue virus [12]. One patient needed mechanical ventilatory support. He also developed neurological manifestations. Transient psychological disturbance is often seen in patients with MIS-C due to COVID-19 [18], and dengue [19].

After consultation with pediatric cardiologists, the patients received treatment with IVIG, methylprednisolone, oral prednisolone, aspirin, clopidogrel, and enoxaparin. All patients recovered with prompt management and were moved to the pediatric ward from the PICU. They were later discharged with advice and follow-up.

## Conclusions

Overlapping outbreaks of SARS-CoV-2 infection and dengue are occurring in some Asian countries. In dengue-endemic countries like Bangladesh, co-infection with COVID-19 is possible and poses a serious challenge and requires timely intervention. In all five cases mentioned here had features of shock, capillary leakage, features of pneumonia, mucocutaneous involvements, variable degree of coagulopathy, altered liver functions and cardiac involvements. Raised inflammatory markers and cardiac enzymes were observed. Cross-reactivity can occur between the antibodies of both viruses, and the similar signs, symptoms, and laboratory findings make the diagnosis harder. On echocardiogram, all patients were found to have coronary arterial dilatations, which was not a documented feature of severe dengue with multi system involvements. In conclusion, the unusual course of severe dengue in these five patients prompted us to look for an explanation. Concomitant severe dengue with MIS-C due to SARS-CoV-2 was considered; alternatively, dengue virus as an unusual etiology for Kawasaki disease was also entertained. Both considerations have not been reported. This increases the chance of missing the diagnosis and delaying the start of appropriate management. We believe this case series may help physicians considering the possibility of co-infection of dengue and MIS-C due to COVID-19, or dengue with unusual etiology for Kawasaki disease rather than focusing on a single disease, in patients with similar presentations.
